# Analysis of the Nursing Effect of Respiratory Critical Illness Based on Refined Nursing Management

This article has been retracted.

**DOI:** 10.1155/2022/6458705

**Published:** 2022-02-08

**Authors:** Wenjuan Shi, Ying Shen, Beilei Zhang, Mengni Jin, Jiale Qian, Xiaoliang Jin

**Affiliations:** Department of Pulmonary and Critical Care Medicine, The First Affiliated Hospital of Soochow University, Jiangsu Province 215000, China

## Abstract

In order to improve the nursing effect of respiratory critical illness, this paper combines the refined nursing method to explore the nursing plan of respiratory critical illness. Moreover, this paper uses the variable control method to explore the effects of nursing management, combines the hospital patient samples to conduct a controlled trial analysis, and conducts sample grouping according to the random grouping method. The patients in the control group are managed by traditional nursing management methods, the patients in the test group are managed by refined nursing management methods, and other conditions are basically the same. In addition, the experiment process variable control is carried out according to the mathematical statistics method, and the reasonable statistics and data processing are carried out. Through the comparison method, we can see that the refined management method proposed in this paper has a good effect in the nursing of respiratory critical illness.

## 1. Introduction

With the advancement of social science and technology, people's quality of life has improved. However, under the development of science and technology, a large amount of pollution is inevitable, and the incidence of some respiratory diseases has greatly increased, becoming one of the diseases with the highest incidence in people [1]. People have grown more aware of their own health concerns as their living conditions have risen, and respiratory ailments have been a focal point in my country's primary disease prevention efforts. It is critical to accomplish illness prevention and treatment as soon as feasible in order to avoid respiratory disorders. Although domestic and international efforts have been committed to the study of the respiratory system in recent years, and different research projects on the respiratory system have been carried out, early detection of respiratory disorders remains a tough direction to overcome [2]. The medical data collected every year has increased tremendously since the dawn of the information age and the acquisition of a big number of medical data, resulting in a huge medical wealth. The stored medical information includes basic inpatient information, long-term/temporary medical advice, electronic medical records, diagnostic information, nursing records, laboratory examinations, imaging examinations, surgical records, transfer records, and patient death information, among other things. Furthermore, individuals are increasingly confronted with a variety of complicated data types, including medical unstructured data, medical semistructured data, and medical structured data. Typical analytic techniques are difficult to utilize to evaluate and mine this complicated kind of data, and traditional approaches are unable of extracting curative aspects from a variety of data formats. As a result, powerful artificial intelligence technology must be used to mine and analyze medical data, NLP technology must be used to extract information from medical unstructured data, and algorithms must be used to examine pathogenic aspects throughout the full medical data set. To advance human medical technology, artificial intelligence technology collects the most important information from a big quantity of medical data [3].

Nursing management is an activity process whose main purpose is to improve nursing quality and work efficiency. The World Health Organization (WHO) pointed out that “nursing management is to improve people's health and to systematically utilize the potential of nurses and other personnel, equipment and social activities.” Hospital nursing management is to study the characteristics of hospital nursing work, find out its regularity, and scientifically plan, organize, control, and coordinate the elements of nursing work, such as personnel, technology, equipment, and information, so as to maximize the nursing system. Optimal operation amplifies the efficiency of the system and provides optimal care for patients. Administrative management, business management, and education management are the three components of nursing management. Nursing administrative management refers to the establishment of a complete and thorough work plan and plan by the nursing organization in order to achieve its established goals, as well as a rational organization established by appropriate people, finances, and materials, using effective leadership methods, and correct and active nursing administration, implementing the nursing organization's incentive method, seeking coordination and communication of opinions among various units and personnel, taking into account the use of time and space, constantly assessing and improving management methods and methods, successfully achieving the nursing organization's overall goals, and placing a high priority on patient care quality. The business and technical management actions carried out to maintain and enhance the efficiency and quality of nursing work are referred to as business management. Nursing laws and regulations, technical specifications, and quality standards, as well as the creation and promotion of new enterprises and technologies, and the organization and direction of nursing research, are all included. Educational management refers to the process of planning and implementing training activities to enhance the quality and professional level of nursing staff at all levels, including nursing student teaching, new nurse preservice training, and on-the-job nurse training and improvement.

With the rapid development of modern science and medical science, various new technologies are widely used in clinical practice, and the transformation of medical nursing models and the renewal of human health concepts, the objects, content, and scope of nursing services are also changing. This change is important for nursing care. Managers put forward new requirements. The traditional parental experience management in the past can no longer keep up with the development needs of nursing disciplines. In the face of new problems that constantly appear in the new era, nursing managers must continue to learn new management ideas and methods if they want to achieve high-level management results. In recent years, people have proposed some new management methods for improving the professional level of nursing and improving the quality of patient care.

This article combines refined nursing management methods to improve the effectiveness of respiratory critical care and provides a theoretical reference for subsequent respiratory critical nursing.

## 2. Related Work

A variety of risk factors can induce ARDS, which can be roughly divided into direct lung injury (pulmonary injury) and indirect lung injury caused by extrapulmonary factors (extrinsic lung injury). Direct lung injury is common in diffuse lung infection, aspiration, and lung contusion. Indirect injuries are common in systemic inflammatory response syndrome (SIRS), metabolic disorders, drug overdose, massive blood transfusion, cardiopulmonary bypass, shock, and so on. If the above two or more risk factors occur, the incidence of ARDS increases significantly. Moreover, the longer the duration of the risk factors, the worse the patient's prognosis. When high-risk factors lasted for 24 h, 48 h, and 72 h, the incidence of ARDS also increased to 76%, 85%, and 93%, respectively [4]. The literature [5] retrospectively analyzed the clinical data of 62 patients with ARDS in the ICU and found that there was no statistical difference in the total mortality of the patients (45.5% and 45%, respectively, *P* > 0.05). However, there were statistical differences between the two groups in terms of ventilator use time and ICU hospitalization time [(7.3 ± 3.8) d vs. (11.5 ± 6.5) d; (9.5 ± 3.2) d vs. (13.6 ± 7.4) d; *P* < 0.05]. According to the comparative analysis of age subgroups, the literature [6] found that the mortality of ARDS patients under 60 years old due to exogenous lung injury was lower than that of the pulmonary injury group (33%, 44%, *P* < 0.05). However, the 7-day mortality rate was higher than that of the exogenous lung injury group (22.7% and 30.8%, respectively, *P* < 0.05). In the over 60 years old group, the 7-day mortality and in-hospital mortality of patients in the extrinsic lung injury group were higher than those in the lung injury group (57.9% vs. 50%; 32.3% vs. 20.5%, *P* < 0.05). The possible reason is that patients with ARDS caused by exogenous lung injury have more complications and are prone to multiple organ dysfunction.

The body's resistance steadily declines with age, and the incidence of ARDS rises as the number of comorbidities rises. The incidence of ARDS in patients aged 60-69 who were hospitalized to the hospital owing to trauma was much greater than that of other age groups, according to the literature [7]. Patients over the age of 80, on the other hand, have the same risk of ARDS as those between the ages of 13 and 19, but the fatality rate of ARDS patients over the age of 80 is much higher. The literature [8] indicated that age > 65 years (area under the ROC curve 0.54) constituted an independent risk factor for mortality in ARDS patients in a retrospective examination of 4397 instances of ARDS patients induced by trauma. The literature [9] conducted a stratified cohort study of 220 ARDS patients and found the mortality rate of patients who were older than 62 years old, the respiratory plateau pressure was greater than 29cmH2O, and PaO2/FiO2 was less than 112 mmHg was significantly increased. The mortality of ARDS patients without the above three risk factors was 12%, while the mortality of patients with the above three risk factors increased to 90%, and there was a statistical difference between the two groups (*P* < 0.001). In the article on predictors of mortality in ARDS, the literature [10] conducted a statistical analysis based on the prognosis of patients and found that the age of the survival group was lower than that of the death group (32.0 ± 11.8 years, 39.1 ± 12.4 years, respectively, *P* = 0.008). However, there are different reports. The literature [11] found that the mortality rate of ARDS patients aged ≥65 years was 51.9%, while the mortality rate of patients under 65 years old was 41.7%. Moreover, there was no statistical difference between the two groups of patients (*P* > 0.05), and no correlation between age and ARDS mortality was found in logistic regression analysis.

After the body is impacted by trauma, severe illness, or other factors, MODS refers to the consecutive functional loss of two or more organs. MODS manifests itself in the lungs as ARDS. According to the literature [12], the incidence of ARDS in the ICU ranges from 10% to 15%, with a death rate of 40% to 50%. Despite the fact that ARDS is characterized by hypoxia and severe respiratory failure, the majority of patients die from MODS. As a result, it is advocated that ARDS be classified as a systemic condition. The incidence of ARDS fatalities attributable to MODS is rising year by year, according to literature [13] study on ARDS meta-analysis, and MODS is without a doubt the most significant risk factor determining the prognosis of severe ARDS patients. The literature [14] conducted a prospective research analysis on 191 patients with confirmed ARDS and found that the deaths of ARDS patients caused by MODS accounted for 77%. Multivariate analysis showed that the number of organ failures ≥ 3 became an independent risk factor for increasing the mortality of patients (OR 11.8; 95% CI: 2.5-55.4; *P* = 0.002). This further confirms that ARDS is a systemic disease.

In the randomized trial study of literature [15], 861 patients were randomly assigned to the two groups with tidal volume of 6 mL/kg and 12 mL/kg. The results showed that the plasmas IL-6 and IL of patients in the low tidal volume treatment group were 6 mL/kg. The level of -8 was significantly lower than that of the 12 mL/kg tidal volume group. Experiments have shown that plasmas IL-6 and IL-8 are closely related to the morbidity and mortality of ARDS patients. Therefore, treatment of ARDS with small tidal volume reduces the inflammation in the body, thereby reducing ARDS death rate. In order to clarify the effect of low tidal volume on the prognosis of mechanical ventilation therapy in patients with ARDS, a study initiated through the Internet showed that treatment with low tidal volume (6.2 ± 0.8 mL/kg) can significantly reduce compared with higher tidal volume (11.8 ± 0.8 mL/kg) mortality in ARDS patients [16]. The best choice of PEEP can not only avoid alveolar damage caused by excessive expansion of alveoli but also prevent alveolar collapse at the end of expiration. The literature [17] showed that at the same time of 5-8 mL/kg small tidal volume ventilation treatment, the static PV curve low turning point pressure increased by 2 cmH2O as the best PEEP, the results compared with conventional ventilation therapy, and the mortality rate of ARDS patients was significantly reduced [17/50 (34%) vs. 25/54 (55.5%), *P* = 0.041)]. Literature [18] also confirmed that small tidal volume and appropriate increase of PEEP can effectively reduce the mortality of ARDS patients. The literature [19] divided 80 patients with ARDS requiring mechanical ventilation into two groups. The low turning point method and the FiO2-PEEP incremental method (PEEP was set by maintaining normal oxygenation goals) were used in PEEP selection, and the patients were treated before the 5th and 12th days. Cytokines (IL-6, IL-8) were significantly lower than the latter, and the oxygenation index on the 12th day was significantly higher than the latter (*P* < 0.05). Mean arterial pressure (MAP) and central venous pressure (CVP) were higher than the former. The impact was small in patients (*P* < 0.05), and complications and average length of stay were lower, with statistical differences (*P* < 0.01). In the literature [20], 549 patients with ARDS requiring mechanical ventilation were randomly divided into the high PEEP group (13.2 ± 3.5 cmH2O) and low PEEP group (8.3 ± 3.2 cmH2O) under the same 6 mL/kg low tidal volume condition. There was no statistical difference in the mortality of the two groups of patients (*P* = 0.48).

## 3. Materials and Methods

All patients enrolled in the study are from January 2019 to 2020 hospital comprehensive ICU inpatients. The patients are randomly divided into a test group and a control group, and the test group implemented meticulous management.

The research content is formulated by the author with reference to similar researches at home and abroad. The collected content includes the patient's gender, age, and various laboratory results when the patient enters the department. The research content includes whether the patient has VAP, the time of mechanical ventilation of the patient, the time of antibiotic use, the length of stay in the ICU, and the pathogen of the sputum culture of the confirmed VAP patient.

Two nurses work together to provide oral care to patients using chlorhexidine nursing solution with a concentration of 0.12 percent in line with normal oral care practices. (2) Subglottic secretions are suctioned. Suctioning of subglottic secretions occurs once per hour. The tracheal cannula and the tracheal cannula have somewhat distinct structures; hence, their procedures are slightly different. To prevent the flushing fluid from leaking into the lungs in patients with tracheal intubation, the balloon pressure should be kept around 25 cmH20 during aspiration, 3-5 mL sterile water should be injected from the flushing tube, and a negative pressure suction device should be connected to the lumen for suction. The procedures described above must be repeated until the suction fluid is clear. The tracheostomy cannula has a flushing tube and a suction tube; so, the flushing tube is continuously filled with sterile water for injection, the suction tube is connected to the negative pressure device, and the operation is continued until the suction liquid is clear, as opposed to the tracheal cannula. (3) Expectoration by vibration: before sputum expectoration, the nasal feeding nutritional solution should be terminated and oxidized aerosol inhalation administered. When the patient expects sputum, he or she sits down. The side lying position is essential for patients who cannot endure it, and the nurse assists in adjusting the patient's posture. The nurse then switches on the expectoration device's switch and counts down 10-20 minutes, depending on the patient's condition. The pace has been lowered to about 30cap/s. The expectoration device is placed near to the patient's back skin and progressively moves upward from the lower lobe of the lung, alternating the lungs. The nurse must be requested to suck sputum after the sputum expectoration, and the patients in the test group must excrete sputum with mechanical vibration twice a day. Other fundamental care practices were the same for all groups of patients, and hand cleanliness was strongly enforced. Sputum is collected and cultured on the day of mechanical ventilation or admission, a chest radiograph is conducted at the bedside, and the chest radiograph is reexamined the following day for mechanically ventilated patients. We use a DRE controllable sputum suction tube or a fiberoptic bronchoscope to retain and remove respiratory secretions in patients who have been on mechanical ventilation for more than 48 hours, and we combine the patient's clinical treatment and clinical manifestations to determine the timing and frequency of sputum culture and send it for examination.

The disease severity classification system must be based on objective physiology and test results parameters and minimize the impact of different treatment measures on patients. The disease severity classification system should be applicable to multiple diseases and easy to use, and most hospitals can obtain the selected parameters. The severity of acute diseases can be assessed by quantifying the degree of abnormality of multiple physiological parameters. For this reason, Knaus proposed APACHE.II, a modified version of APACHE in 1985. The highest score of APACHE is 71 points. The higher the score obtained by the patient, the more serious the disease. It can objectively formulate and revise patient's treatment plan and nursing measures through the evaluation of the condition of ICU patients, the prediction of underlying diseases, and the mortality rate. Moreover, it provides a scientific and objective basis for improving the quality of medical care, improving the effect of treatment, rationally using medical resources, and determining the best time to discharge or choose the time for treatment. The APACHEII score can be used for the comparison of patients with a single disease, and it can also be used for the evaluation of patients with mixed diseases. The APACH II score is also applicable to critically ill patients in general wards. Since the advent of the APACHII scoring system, it has been recognized by the medical community for its simplicity, reliability, and ease of data collection. It has become a scoring system commonly used in ICUs worldwide. Therefore, this experiment mainly uses this score to verify whether the differences between the groups are comparable, which has a high degree of credibility.

The test and control groups' nursing staffs were all professionally qualified nursing staff in the undergraduate room. Nursing tasks that need nursing personnel (such as patient bedside elevation, dental care, and sputum retention) are universally taught and standardized. The tasks that need the doctor's collaboration (such as cleaning the effusion on the capsule, vibration, and expectoration) are completed with the laboratory staff's assistance to guarantee that the patients get consistent therapy.

All the collected cases of the patients enrolled in the group were collected by the experimenters themselves. From the time the patient is enrolled, it is necessary to observe the patient's condition every day, collect data, and keep the laboratory results and scores of the patients when they are enrolled in the group. When the patient is transferred out, discharged from the hospital, or died, relevant data needs to be retained again. The collected data is unified into the Microsott Excel table and reviewed.

## 4. Result

The incidence of ventilator-associated pneumonia in the test group was 18.18%, and the incidence of ventilator-associated pneumonia in the control group was 35.13%. Compared with the control group, the incidence of VAP in the test group was significantly lower, and the difference was statistically significant (*P* < 0.05). Through statistics of the survival rates of patients at 28 days and 90 days, it is found that the 28-day test group has a mortality rate of 12.73%, and the control group 7 has a mortality rate of 18.92%. The results of statistical analysis show that there is no statistically significant difference in 28-day mortality between the two groups (*P* > 0.05). At 90 days, the mortality rate of 55 patients in the test group is 23.64%, and that of the control group is 31.08%. Through statistical analysis of the results, it can be seen that the 90-day mortality difference between the two groups of patients is not statistically significant (*P* > 0.05). The specific results are shown in Table 1.

By analyzing the treatment effect of the two groups of patients, it is found that the mechanical ventilation time of the test group is shorter than that of the control group, and the difference is statistically significant (*P* < 0.05). Moreover, the antibiotic use time in the test group is shorter than that in the control group, and the difference is statistically significant (*P* < 0.05). The ICU stay time of the test group is shorter than that of the control group, and the difference is statistically significant (*P* < 0.05). The results are shown in Tables 2–4.

This article counts the comprehensive evaluation of respiratory critical nursing in the test group and the control group, and the results are shown in Table 5.

It can be seen from the above studies that the comprehensive evaluation of the experimental group is significantly higher than that of the control group. On this basis, patient satisfaction statistics are performed, and the results are shown in Table 6.

It can be seen from the above research that the refined management method proposed in this paper has a good effect in the nursing of respiratory critical illness.

## 5. Analysis and Discussion

Current medical and nursing research is focused on how to avoid VAP. The Institute for Healthcare Improvement (IHI) presented a cluster management plan for mechanically ventilated patients that included four core measures: elevating the bed, waking up daily, avoiding stomach ulcers, and preventing deep vein thrombosis. Furthermore, each of the approaches has been shown to enhance the prognosis of patients who are mechanically ventilated. However, as research has progressed, it has been shown that the clustering program still has flaws in terms of preventing VAP, particularly in terms of managing oropharyngeal flora and subglottic secretions. Furthermore, certain novel approaches have been shown to minimize the prevalence of VAP. In terms of the four main clustering measures, this research delivers patients' chlorhexidine oral care and subglottic secretions to attract and vibrate sputum, which not only inhibits oropharyngeal flora colonization and reproduction but also increases sputum release from the lungs. The incidence of VAP in the test group has reduced compared to the control group following the adoption of clustering measures and improved management, as shown in the above experimental data, and the difference is statistically significant. The test group's mechanical ventilation time, antibiotic usage time, and ICU stay duration are all reduced when compared to the control group, and the result is statistically significant. This demonstrates that implementing clustering strategies and attentive monitoring of mechanically ventilated patients may not only minimize the incidence of VAP but also increase the therapeutic impact. However, when the 28-day and 90-day survival rates of the two groups of patients are compared, it is discovered that there is no substantial difference in mortality between the two groups. It is possible that the explanation for this is that the number of cases included was inadequate, and the treatment effects obtained in each department after patients were moved from the ICU were different. The onset of VAP can be summarized as two reasons for the increased chance of pathogen invasion and the weakening of the patient's immune mechanism. The former includes damage to the respiratory barrier caused by artificial airways, aspiration of colonized pathogens in the oropharynx, contamination of the ventilator pipeline, long-term mechanical ventilation, and even crossinfection of medical staff. The latter includes elderly patients, malnutrition, impaired systemic immune mechanisms, retention of subglottic secretions, migration of gastrointestinal flora, and antibiotic abuse. Next, we elaborate on the etiology and pathogenesis of VAP.

Patients who are admitted to the ICU and undergo mechanical ventilation are mainly elderly patients. Due to the older age of the patient, the physiological functions and various bodily functions of the elderly have declined. In particular, the elderly usually has basic diseases such as hypertension, coronary heart disease, diabetes, and acute and chronic renal failure. Therefore, such patients are more likely to develop VAP. The United States Hospital Infection Detection Organization lists ages older than 70 as a risk factor.

Due to the severe condition of mechanically ventilated patients, such patients cannot eat through the stomach. Generally, enteral nutrition or even parenteral nutrition is used to provide patients with essential amino acids and other nutrients. Moreover, mechanically ventilated patients generally have different degrees of nutritional intake disorder, showing a negative nitrogen balance. The body's high catabolism state increases its sensitivity to bacteria. Therefore, the conditional pathogenic bacteria and fungi that exist in the human body can accelerate the reproduction and cause infection due to the patient's own hypoproteinemia.

Mechanically ventilated patients in the ICU are often critically ill or after major surgery. The patients are generally in a state of consciousness disorder, shock, coma, long-term bed rest, and multiple organ failure. This leads to an increase in the probability of patients being infected, the use of broad-spectrum antibacterial drugs, or the use of antibacterial drugs in combination. The use of broad-spectrum antibacterial drugs and combined use of antibacterial drugs will change the structure and proportion of the patient's normal flora, leading to the emergence of fungal infections and drug-resistant bacteria, multiple infections, and refractory VAP.

Patients who are mechanically ventilated are usually given parenteral nourishment by central vein or enteral nutrition via gastric tube since they are unable to consume by mouth. Long-term parenteral nourishment induces gastric mucosa atrophy and inhibits its protective role, allowing germs to grow and spread more readily, exacerbating lung infections. Acid inhibitors are often used in the ICU to avoid stress ulcers in critically sick and surgical patients by inhibiting gastric acid production and reducing gastric acid invasion of the stomach mucosa. However, when gastric acid output decreases, the pH value in the stomach rises, gastric acid's bactericidal function is decreased, and bacteria are more prone to colonize and grow in the stomach. Furthermore, owing to the indwelling of the gastric tube, the function of the lower esophageal sphincter is impaired while employing enteral feeding, which readily causes reflux and aspiration of the stomach contents. At the same time, aspirated things into the lungs may readily induce lung infections owing to the enormous number of bacteria in the stomach.

The cluster management measures of ventilator-associated pneumonia have been widely used in clinical practice. The four basic measures are raising the head of the bed, waking up daily, preventing peptic ulcers, and preventing deep vein thrombosis, and each measure has evidence that it can improve the prognosis of mechanically ventilated patients. However, with the in-depth research on ventilator-associated pneumonia, it has been found that the clustering program can still be improved in the prevention of VAP, especially in the management of oropharyngeal flora and subglottic secretions. Moreover, recent studies have shown that many new measures can further reduce the incidence of VAP in patients with prolonged mechanical ventilation. Therefore, adding chlorhexidine oral care, suction of subglottic secretions, and vibrating sputum on the basis of cluster management can reduce the possibility of secondary infection, thereby reducing the incidence of VAP in patients with mechanical ventilation, shortening the time of mechanical ventilation, ICU stay time, and antibiotic use time, which is worthy of clinical promotion. Pathogenic bacteria in VAP patients are mostly Gram-negative bacilli, according to an investigation of pathogenic bacteria in VAP patients. The most common species is Pseudomonas aeruginosa, whereas Gram-positive bacteria are mostly Staphylococcus aureus and fungi are the least common. The most prevalent infections in ICU are Pseudomonas aeruginosa, Acinetobacter baumannii, and Staphylococcus aureus. As a consequence, while treating VAP patients with antibacterial medicines, clinical and drug sensitivity outcomes should be considered. The test group had no meaningful influence on patient survival rates at 28 and 90 days, according to the research. It is possible that the explanation for this is because the number of cases included was inadequate, and the treatment effects obtained in various departments after patients are moved from the ICU varied. The whole ICU staff is, of course, the most critical aspect in the overall prevention of VAP. VAP can only be properly averted when physicians and nurses work together to carefully apply these precautions.

## Figures and Tables

**Table 1:** The incidence of VAP and the survival rate of patients in the two groups.

	Test group	Control group
VAP incidence	18.16%	35.12%
28-day mortality	12.71%	18.90%
90-day mortality	23.61%	31.06%

**Table 2:** Mechanical ventilation time (D).

No.	Test group	Control group	No.	Test group	Control group
1	9.50	9.41	13	7.46	13.44
2	8.37	8.79	14	4.43	6.17
3	6.51	5.55	15	9.11	6.09
4	11.70	5.35	16	5.16	12.71
5	5.50	12.85	17	4.81	13.37
6	11.87	5.35	18	9.61	13.53
7	9.09	15.06	19	9.69	11.26
8	9.48	10.85	20	9.21	13.58
9	8.19	14.78	21	9.01	5.05
10	7.97	10.90	22	9.93	7.96
11	4.90	7.12	23	4.55	10.96
12	6.09	8.73			

**Table 3:** Antibiotic use time (D).

No.	Test group	Control group	No.	Test group	Control group
1	5.02	10.65	13	4.45	4.36
2	11.97	4.09	14	3.71	5.43
3	7.67	14.92	15	8.30	15.56
4	4.24	10.45	16	5.61	3.90
5	4.09	5.03	17	3.94	11.45
6	11.80	4.58	18	3.20	8.60
7	6.21	15.50	19	5.52	9.02
8	11.26	11.43	20	4.24	13.62
9	6.23	3.08	21	4.66	15.39
10	4.59	4.56	22	2.65	12.14
11	5.67	9.27	23	8.65	2.92
12	10.32	8.54			

**Table 4:** ICU residence time (D).

No.	Test group	Control group	No.	Test group	Control group
1	10.00	25.38	13	9.44	17.15
2	18.40	20.58	14	21.36	22.03
3	11.50	26.31	15	6.86	22.83
4	9.95	26.69	16	8.15	11.65
5	16.69	18.26	17	17.33	10.42
6	20.09	14.37	18	14.56	20.79
7	7.17	14.45	19	9.98	27.48
8	7.90	23.12	20	20.30	26.93
9	11.22	11.30	21	15.55	12.91
10	7.72	20.62	22	19.58	12.68
11	9.13	21.82	23	13.49	17.71
12	20.58	26.05			

**Table 5:** Comprehensive evaluation of nursing effect.

No.	Test group	Control group	No.	Test group	Control group
1	88.45	86.73	13	94.98	85.09
2	88.21	87.27	14	89.34	79.53
3	89.87	91.15	15	92.34	81.40
4	95.82	76.80	16	96.28	79.23
5	94.68	78.21	17	84.43	89.39
6	83.84	72.98	18	96.15	94.86
7	83.08	90.34	19	92.82	86.85
8	94.07	89.92	20	85.12	87.70
9	91.22	76.97	21	96.95	77.07
10	92.07	92.43	22	90.59	75.05
11	94.71	78.37	23	96.36	71.67
12	86.42	72.76			

**Table 6:** Statistical table of patient satisfaction.

No.	Test group	Control group	No.	Test group	Control group
1	96.45	90.50	13	96.36	91.87
2	97.73	92.71	14	94.77	83.47
3	93.59	90.59	15	93.78	88.98
4	91.24	82.49	16	91.47	76.63
5	95.76	86.12	17	97.05	85.97
6	91.90	92.87	18	91.05	77.05
7	95.88	91.67	19	94.62	77.33
8	94.96	86.28	20	97.57	76.25
9	97.80	83.27	21	97.03	87.30
10	93.21	89.37	22	92.71	85.01
11	95.83	87.10	23	93.27	82.20
12	97.25	87.63			

## Data Availability

The data used to support the findings of this study are included within the article.
